# Diagnostic Value and Clinical Performance of Cardiac Ultrasound in Patients with Chronic Heart Failure with Hypertension

**DOI:** 10.1155/2022/4238284

**Published:** 2022-05-05

**Authors:** Punan Li, Xiaoli Zhang

**Affiliations:** Cardiac Ultrasound Group, Department of Ultrasound Medicine, Jincheng People's Hospital, Jincheng 048000, Shanxi Province, China

## Abstract

**Objective:**

To assess the diagnostic value and clinical performance of cardiac ultrasound in patients with chronic heart failure and hypertension.

**Methods:**

In this prospective study, between August 2017 and January 2020, 50 patients with chronic heart failure and hypertension were recruited and assigned to the study group and 50 healthy individuals during the same period after physical examinations were included in the control group. Cardiac ultrasound examinations were performed on the participants, and the results were compared and analyzed.

**Results:**

The study group had a higher left ventricular end-diastolic diameter (LVEDD), left ventricular end-systolic diameter (LVESD), left ventricular ejection fraction (LVEF), and late diastolic peak flow velocity (A wave) and showed lower early diastolic peak flow velocity (E wave) and late diastolic peak flow velocity/lower early diastolic peak flow velocity (E/A) ratio levels than in the control group. The study group had 15 patients with grade I cardiac function (ultrasound detection rate of 100%), 18 patients with grade II cardiac function (ultrasound detection rate of 100%), and 17 patients with grade III cardiac function (ultrasound detection rate of 100%). Grade I cardiac function patients showed the lowest LVEDD, LVESD, and E/A and the highest LVEF than grade II patients, followed by grade III patients. The study group showed higher LVEF and echocardiographic estimation of the pulmonary arterial systolic pressure (PASP) and lower right ventricular lateral wall systolic excursion velocity and tricuspid annular plane systolic excursion (TAPSE) than the control group. Chronic heart failure with hypertension was associated with high levels of right atrial total emptying volume (RAVIt), right atrial passive emptying volume (RAVIp), right atrial active emptying volume (RAVIa), and right atrial active emptying fraction (RAVIaEF) and low levels of right atrial total emptying fraction (RAVItEF) and right atrial passive emptying fraction (RAVIpEF) versus the healthy status (all *P* < 0.05).

**Conclusion:**

Cardiac ultrasound is a noninvasive operation with low cost, high repeatability, and accurate detection, which can identify right heart function impairment at an early stage, assist clinical treatment, and improve patient prognosis, so it is worthy of promotion and application.

## 1. Introduction

Chronic heart failure (CHF) is a common clinical complication of cardiovascular diseases [1], which refers to the failure of normal myocardial contraction elicited by various diseases to provide sufficient blood for normal metabolism [2]. It is the end stage of diverse cardiovascular diseases such as coronary artery disease and cardiomyopathy and is mostly associated with hypertension, aortic stenosis, pulmonary hypertension, pulmonary stenosis, heart valve closure insufficiency, left and right heart or arteriovenous shunt congenital cardiovascular diseases such as a septal defect, and arteriovenous insufficiency, among which primary hypertension is considered one of the most common pathogenic factors in patients with CHF [3, 4]. Long-term substandard blood pressure control may lead to left ventricular hypertrophy, ventricular diastolic function degradation, and ultimately cardiac insufficiency, and the treatment efficacy of right heart failure is also unsatisfactory [5]. The disease is highly prevalent in the elderly population, with an increasing incidence in recent years, which is a current research hotspot [6]. Research has reported a comparable survival rate for patients with multiple cause CHF and malignant neoplastic diseases, with a high mortality rate exceeding 50%. Thus, an early and accurate diagnosis of multiple cause CHF and active treatment contributes to improving the prognosis and the quality of life of patients [7]. Cardiac ultrasound has been widely used in the diagnosis of CHF as a safe and reliable diagnostic technique [8]. Previously, single indices such as left ventricular ejection fraction (LVEF) were used for the evaluation of CHF, but the accuracy of the assessment remains unfavorable [9]. Considering the concomitance of abnormal systolic and diastolic functions of the heart with alterations in a cardiac structure, a comprehensive evaluation of cardiac function using multiple indices is considered more reliable [10]. Studies have pointed out that cardiac ultrasound yields a promising value in the diagnosis of various clinical diseases with a well-recognized advantage in diagnosing CHF; however, further investigation is required regarding its value in the diagnosis of multiple cause CHF [11, 12]. Accordingly, this study was conducted to assess the diagnostic value and clinical performance of cardiac ultrasound in patients with chronic heart failure and hypertension and to provide effective references for future clinical diagnosis and treatment. The results are as follows.

## 2. Materials and Methods

### 2.1. Baseline Data

In this prospective study, between August 2017 and January 2020, 50 patients with chronic heart failure and hypertension were recruited and assigned to the study group, and 50 healthy individuals during the same period after physical examinations were included in the control group. The study was approved by the Ethics Committee of the Jincheng People's Hospital, No. 201JC8/71.

### 2.2. Inclusion and Exclusion Criteria

Inclusion criteria were as follows: ① patients who met the diagnostic criteria for CHF in the Chinese heart failure diagnosis and treatment guidelines 2018; ② patients who met the diagnostic criteria for primary hypertension in the Chinese guidelines for the prevention and treatment of hypertension (2018 revision); and ③ patients who provided written informed consent and voluntarily participated in the study.

Exclusion criteria were as follows: ① patients with incomplete clinical data; ② patients with severe dysfunction of the liver, kidney, and other organs or malignant tumors; and ③ patients with congenital mental retardation or mental illness.

## 3. Methods

Ultrasound Doppler for cardiac ultrasound diagnosis was performed in all eligible participants, using the PHILIPS EPIQ7C whole-body application ultrahigh-end cardiac ultrasound sonographer [13] with the phased-array probe, and the probe frequency was set to 2.5–4.0 MHz. With the patient in the prone position, conventional ultrasound results were obtained by continuous scanning of the cardiac structures. The overall morphology and structures of the heart were observed using the two-dimensional cardiac ultrasound images, the orientation of the sampling line was determined on the basis of M-mode echocardiography, and the activity of the upper cardiac structures was observed and recorded in detail. The LVEF was monitored by the biplane Simpson method, and the diastolic forward bimodal flow spectrum was examined using the apical four-chamber views and two-chamber views, and the early peak diastolic flow velocity and late peak diastolic flow velocity were recorded. The ratios of early diastolic peak flow velocity and late diastolic peak flow velocity were calculated in detail. After obtaining LVEF, right ventricular lateral wall systolic displacement velocity, TAPSE, and PASP, the values of right atrial total emptying volume (RAVIt), right atrial passive emptying volume (RAVIp), and right atrial active emptying volume (RAVIa) were calculated using the 3DQA system, and the values of right atrial total emptying fraction (RAVItEF), right atrial passive emptying fraction (RAVIpEF), and right atrial active emptying fraction (RAVIaEF) could also be obtained, each of which were calculated by taking the mean value of the data of 3 cardiac cycles.

### 3.1. Outcome Measure

The LVEDD, LVESD, LVEF, early diastolic peak flow velocity (E wave), late diastolic peak flow velocity (A wave), and the E/A ratio were recorded and compared between the two groups. The data of the indexes in the observation group were compared under different cardiac functional status classifications. LVEF, right ventricular lateral wall systolic displacement velocity, TAPSE, and pulmonary arterial systolic pressure (PASP) were recorded. PASP was calculated by measuring the transvalvular pressure difference using the tricuspid systolic reverse flow spectrum. The values of RAVIt (RAVIt = RAVImax–RAVImin), RAVIp, RAVIa, RAVItEF, RAVIp EF (RAVIp EF = RAVIp/RAVImax), and RAVIaEF (RAVIaEF = RAVIa/RAVIpre) were calculated and compared.

RAVIa indicates the right atrial pumping function, and the peak right atrial filling rate in systole (dv/dt S, representing the storage function of the right atrium), peak right atrial emptying rate in early diastole (dv/dt E, representing the ductal function of the right atrium), and peak right atrial emptying rate in late diastole (dv/dt A, representing the pumping function of the right atrium) were recorded according to the obtained right atrial volume change rate curve.

### 3.2. Statistical Analysis

SPSS22.0 software was used to process the data. The count data were expressed as (n (%)) and processed using the chi-square test, and the measurement data were expressed as (‾*x* ± *s*) using the *t*-test. Comparisons between multiple groups were conducted using the one-way method of analysis, and two-by-two comparisons were performed using the LSD-t-test. Differences were considered statistically significant at *P* < 0.05.

## 4. Results

### 4.1. Baseline Data

The baseline features of the eligible patients in the study group (29 males and 21 females, mean age of (55.37 ± 11.67) years, mean BMI of (24.01 ± 2.14) kg/m^2^, course of hypertension of (8.13 ± 2.37) years, and course of CHF of (6.05 ± 1.68) years) were comparable with those of the included healthy subjects (26 males and 24 females, mean age of (55.29 ± 11.84) years, mean BMI of (23.68 ± 2.57) kg/m^2^, course of hypertension of 0 years, and course of CHF of 0 years) (*P* > 0.05) (Table 1).

### 4.2. Conventional Ultrasound

The LVEDD, LVESD, LVEF, and A wave of the study group were (54.88 ± 8.67, 27.92 ± 3.67, 59.76 ± 6.13, and 78.09 ± 10.07), which were significantly higher than those of the control group (51.09 ± 7.81, 25.58 ± 3.53, 55.84 ± 9.46, and 68.16 ± 12.21). The E wave and the E/A ratio of the study group were markedly lower than those of the control group (56.56 ± 12.54 and 0.71 ± 0.99 vs. 82.58 ± 11.25 and 1.35 ± 0.74, respectively) (*P* < 0.05) (Table 2).

### 4.3. Cardiac Function

#### 4.3.1. Assessment of Cardiac Functional Grading

The study group had 15 patients with grade I cardiac function (ultrasound detection rate of 100%), 18 patients with grade II cardiac function (ultrasound detection rate of 100%), and 17 patients with grade III cardiac function (ultrasound detection rate of 100%).

#### 4.3.2. Cardiac Function Data under Cardiac Functional Grading

The LVEF, LVEDD, LVESD, and E/A of grade I patients were 59.41 ± 7.53, 42.37 ± 5.56, 48.21 ± 6.45, and 10.21 ± 4.21; those of grade II patients were 54.21 ± 6.14, 51.21 ± 6.42, 53.65 ± 7.53, and 12.56 ± 4.55; and those of grade III patients were 47.43 ± 6.17, 58.68 ± 7.21, 59.69 ± 8.21, and 17.51 ± 5.12. Grade I cardiac function patients showed the lowest level of LVEDD, LVESD, and E/A and the highest level of LVEF than grade II patients, followed by grade III patients (*P* < 0.05) (Table 3).

### 4.4. Right Atrial Structure

#### 4.4.1. Conventional Ultrasound Results

The LVEF, RASP, right ventricular lateral wall systolic excursion velocity, and TAPSE of the study group were 59.76 ± 6.13, 47.98 ± 3.84, 12.23 ± 2.19, and 16.15 ± 2.87 and those of the control group were 55.84 ± 9.46, 28.35 ± 5.78, 18.56 ± 3.56, and 20.54 ± 4.61. (*P* < 0.05) (Table 4).

### 4.5. Right Atrial Structure Ultrasound Results

The RAVIt, RAVIp, RAVIa, RAVIaEF, RAVItEF, and RAVIpEF of the study group were 18.94 ± 4.79, 10.23 ± 3.88, 6.21 ± 2.45, 37.12 ± 6.13, 43.54 ± 4.18, and 34.28 ± 4.03 and those of the control group were 12.45 ± 2.56, 8.68 ± 2.42, 4.15 ± 1.93, 35.18 ± 5.12, 56.37 ± 5.25, and 45.39 ± 3.61. Chronic heart failure with hypertension was associated with high levels of RAVIt, RAVIp, RAVIa, and RAVIaEF and low levels of RAVItEF and RAVIpEF versus the healthy status (all *P* < 0.05) (Table 5).

## 5. Discussion

Chronic heart failure refers to the inability of the myocardium to contract properly and provide sufficient blood for normal metabolism to satisfy the needs of the body. Primary hypertension is one of the most common factors in the development of CHF [14]. It has been reported that the current survival rate of CHF with multiple causes is comparable to that of patients with malignant neoplastic diseases, with a high mortality rate exceeding 50% [15]. However, conventional diagnosis fails to provide a comprehensive analysis of the cardiac function, resulting in a high risk of misdiagnosis and underdiagnosis, along with the invasiveness of many examinations, which prevents desirable diagnostic results [16, 17]. Ultrasound technology has been widely used in clinical practice, and cardiac ultrasound provides a comprehensive evaluation of the cardiac function by effectively displaying detailed information such as cardiac data and blood flow data of the examined subjects. The use of cardiac ultrasound to perform effective examinations in patients with hypertension and CHF can accurately determine the myocardial lesions, cardiac atrioventricular cavity size, ventricular wall thickness and septal damage, and other relevant indicators, which facilitate the diagnosis and treatment of the disease [18]. It has been shown that cardiac ultrasound, as an important modality for diagnosing the cardiac function, features benefits such as less damage, simplicity of operation, and repeatability, which provide higher sensitivity versus electrocardiographic results and remarkably improve the accuracy of disease diagnosis [19, 20].

In the present study, the diagnosis of hypertensive left ventricular hypertrophy with left heart failure was performed by cardiac ultrasound. The cardiac ultrasound allows the observation of cardiac blood flow as well as cardiac fluctuations and facilitates the clinician's judgment of the patient's myocardial lesions, cardiac atrial wall thickness, and ventricular chamber size. Cardiac ultrasound features advantages such as high reproducibility, noninvasiveness, and high sensitivity compared with traditional electrocardiography, especially for atrial enlargement and early ventricular structural changes. In addition, cardiac ultrasound diagnosis presents dynamic changes in patients with hypertensive left ventricular hypertrophy with left heart failure, which improve the accuracy of clinical diagnosis and facilitate clinicians to observe the structure of patients' heart chambers, which is of high diagnostic value for hypertensive left ventricular hypertrophy with left heart failure.

The results of the current study showed higher LVEDD, LVESD, and LVEF and lower *E* wave and E/A results; moreover, grade I cardiac function patients showed the lowest level of LVEDD, LVESD, and E/A and the highest level of LVEF than grade II patients, and then grade III patients. Research has demonstrated that cardiac ultrasound is considered a key diagnostic modality for the cardiac function, with the advantages of less damage, simpler operation, and repeatability, which contribute to enhance the accuracy of disease diagnosis. The results of the present study also confirmed the accuracy of the examinations of the patients' cardiac function, which was similar to the previous research results. Furthermore, the study group herein outperformed the control group in terms of LVEF, RASP, right ventricular lateral wall systolic excursion velocity, and TAPSE. Chronic heart failure with hypertension in the present study was associated with high levels of RAVIt, RAVIp, RAVIa, and RAVIaEF and low levels of RAVItEF and RAVIpEF versus the healthy status. In the present study, the study group had elevated RAVIt and decreased RAVItEF compared to the control group. During the increment of pulmonary artery pressure, the right atrial volume also enlarges to ensure the injection of blood volume into the right ventricle, but the total emptying capacity is diminished, indicating changes in the right atrial structure in the advanced stage which results in the diminished RAVItEF. The increase of RAVIp and decrease of RAVIpEF indicate that with the increase of right ventricular pressure, the resistance of right atrial inflow into the right ventricle increases, which leads to the decrease of right atrial ductal capacity. The RAVIa and RAVIaEF of the study group were significantly higher than those of the control group, suggesting a compensatory increase in right atrial myocardial capacity in the early stage of elevated pulmonary artery pressure; however, the progressive increase in pulmonary artery pressure causes a loss of the compensatory myocardial contractile function and leads to a reduced right atrial pump function in the chronic heart failure group. Thus, a lower overall right atrial ejection fraction and a higher right atrial volume index are indicative of abnormal right atrial function.

The hemodynamic indexes are the most direct reflection of the cardiac function, in which LVSP and the maximum rate of increase of left intraventricular pressure can determine the systolic performance, and LVEDP and the maximum rate of decrease of the left intraventricular pressure together determine the diastolic performance. The addition of the Shenfu injection to the conventional western medicine treatment provides the effect of restoring yang, relieving deficit, benefiting qi, and removing heat. The Shenfu injection solution is a compound drug, and it is mainly composed of red ginseng and Aconiti Lateralis Radix Praeparata. It is mainly used to treat palpitation, coughing, stomach pain, diarrhea, and paralysis caused by Yang deficiency and Qi deficiency. The Shenfu injection solution significantly improves noninvasive hemodynamic indices in the hearts of patients with chronic systolic heart failure, increases output and cardiac output per beat, decreases peripheral vascular resistance, increases left ventricular ejection fraction, and lowers plasma B-type brain natriuretic peptide concentration. The limitation of this study lies in the absence of testing of diagnostic efficacy and the sensitivity and specificity of ultrasound diagnosis, which will be further investigated in the future.

## 6. Conclusion

Cardiac ultrasound is a noninvasive operation with low cost, high repeatability, and accurate detection, which can identify right heart function impairment at an early stage, assist clinical treatment, and improve patient prognosis, so it is worthy of promotion and application.

## Figures and Tables

**Table 1:** Comparison of baseline data ($\bar{\text{x}}$ ± *s*).

Groups	Gender		Age	BMI	Course of hypertension	Course of CHF
	Male	Female				
Study group	29	21	55.37 ± 11.67	24.01 ± 2.14	8.13 ± 2.37	6.05 ± 1.68
Control group	26	24	55.29 ± 11.84	23.68 ± 2.57	0	0
t	-	-	0.340	0.698	-	-
P	-	-	0.973	0.487	-	-

**Table 2:** Comparison of conventional ultrasound results ($\bar{\text{x}}$ ± *s*).

Groups	n	LVEDD (mm)	LVESD (mm)	LVEF (%)	A wave (%)	E wave (%)	E/A (%)
Study group	50	54.88 ± 8.67	27.92 ± 3.67	59.76 ± 6.13	56.56 ± 12.54	78.09 ± 10.07	0.71 ± 0.99
Control group	50	51.09 ± 7.81	25.58 ± 3.53	55.84 ± 9.46	82.58 ± 11.25	68.16 ± 12.21	1.35 ± 0.74
t	-	2.297	3.249	2.459	10.921	4.436	3.661
P	-	0.024	0.002	0.016	<0.01	<0.01	<0.01

**Table 3:** Assessment of cardiac functional grading of the study group ($\bar{\text{x}}$ ± *s*).

Groups	n	LVEDD (mm)	LVESD (mm)	LVEF (%)	E/A (%)
Grade I	15	42.37 ± 5.56	48.21 ± 6.45	59.41 ± 7.53	10.21 ± 4.21
Grade II	18	51.21 ± 6.42^a^	53.65 ± 7.53^a^	54.21 ± 6.14^a^	12.56 ± 4.55^a^
Grade III	17	58.68 ± 7.21^ab^	59.69 ± 8.21^ab^	47.43 ± 6.17^ab^	17.51 ± 5.12^ab^
F		7.360	3.880	3.784	2.681
P		<0.01	<0.01	<0.01	<0.01

Compared with grade I, ^a^*P* < 0.01 and compared with grade II, ^b^*P* < 0.0.

**Table 4:** Conventional ultrasound results ($\bar{\text{x}}$ ± *s*).

Groups	n	RAVIt (ml/m^2^)	RAVIp (ml/m^2^)	RAVIa (ml/m^2^)	RAVItEF (%)	RAVIpEF (%)	RAVIaEF (%)
Study group	50	18.94 ± 4.79	10.23 ± 3.88	6.21 ± 2.45	43.54 ± 4.18	34.28 ± 4.03	37.12 ± 6.13
Control group	50	12.45 ± 2.56	8.68 ± 2.42	4.15 ± 1.93	56.37 ± 5.25	45.39 ± 3.61	35.18 ± 5.12
t	-	8.450	2.397	4.670	13.519	14.520	1.718
P	-	<0.001	0.019	<0.001	<0.001	<0.001	0.049

**Table 5:** Comparison of structural ultrasound results ($\bar{\text{x}}$ ± *s*).

Groups	n	RAVIt (ml/m^2^)	RAVIp (ml/m^2^)	RAVIa (ml/m^2^)	RAVItEF (%)	RAVIpEF (%)	RAVIaEF (%)
Study group	50	18.94 ± 4.79	10.23 ± 3.88	6.21 ± 2.45	43.54 ± 4.18	34.28 ± 4.03	37.12 ± 6.13
Control group	50	12.45 ± 2.56	8.68 ± 2.42	4.15 ± 1.93	56.37 ± 5.25	45.39 ± 3.61	35.18 ± 5.12
t	-	8.450	2.397	4.670	13.519	14.520	1.718
P	-	<0.001	0.019	<0.001	<0.001	<0.001	0.049

## Data Availability

All data generated or analyzed during this study are included in this article.
